# The Prediction Value of D-Dimer on Prognosis in Intensive Care Unit among Old Patients ( ≥65 Years): A 9-Year Single-Center Retrospective Study of 9261 Cases

**DOI:** 10.1155/2022/2238985

**Published:** 2022-09-22

**Authors:** Hui Lian, Huacong Cai, Hongmin Zhang, Xin Ding, Xiaoting Wang, Shuyang Zhang

**Affiliations:** ^1^Department of Health Care, Peking Union Medical College Hospital, Chinese Academy of Medical Sciences and Peking Union Medical College, Beijing, China; ^2^Department of Hematology, Peking Union Medical College Hospital, Chinese Academy of Medical Sciences and Peking Union Medical College, Beijing, China; ^3^Department of Critical Care Medicine, Peking Union Medical College Hospital, Chinese Academy of Medical Sciences and Peking Union Medical College, Beijing, China; ^4^Department of Cardiology, Peking Union Medical College Hospital, Chinese Academy of Medical Sciences, Beijing 100730, China

## Abstract

**Background:**

D-dimer (DD) has been indicated as a potential indicator due to its connection with the prognosis of the COVID-19 pandemic. Aging is linked to elevated DD levels in coagulation activation. However, few studies have investigated the correlation of DD with prognosis, especially in the old population. Therefore, this study aims **at** investigat**ing** the correlation of DD with prognosis in shock and perioperative populations over 65 years of age.

**Methods:**

We analyzed 9261 old patients admitted to intensive care units (ICUs) with either confirmed shock or in perioperative period of high-risk surgery, with 8813 of them had DD levels determined on admission. In-hospital mortality, length of ICU stay and ventilation time (VT) associated variables were assessed using generalized linear models.

**Results:**

Although DD levels had no positive correlations with in-hospital mortality (RR, 1.006; 95% CI, 0.998-1.014) and length of ICU stay (RR, 1.012; 95% CI, 0.997-1.028) in Model 3, they were strongly correlated with VT (RR, 1.577; 95% CI, 1.024-2.064). Higher DD levels in females (RR, 1.804; 95% CI, 1.116-2.602), those who used antibiotics (RR, 1.736; 95% CI, 1.092-2.453), those with surgery (RR, 1.640; 95% CI, 1.273-2.114), and those with shock (RR, 1.740; 95% CI, 1.001-2.687) had stronger correlation with longer VT than the counterparts. While patients who were between 65 and 74 years old (RR, 1.023; 95% CI, 1.003–1.043), with no use of antibiotics (RR, 1.007; 95% CI, 1.001–1.013) nor shock (RR, 1.011; 95% CI, 1.002–1.021), but had undergone surgical procedures (RR, 1.030; 95% CI, 1.012–1.048) were correlated with a longer ICU length of stay.

**Conclusion:**

DD levels at ICU admission are highly related to increased VT and length of ICU stay in the old population with either confirmed shock or after high-risk surgery, indicating the strong potential of DD as a marker with prognostic utility for all ICU patients in the future.

## 1. Introduction

The proportion of old patients ( ≥65 years) in the Intensive Care Unit (ICU) has significantly increased as a result of population aging [1–3]. Aging leads to deterioration of organ function, which is usually correlated with imbalances in oxygen supply and demand, endothelial dysfunction, and coagulopathy [4]. D-dimer (DD), as a fibrin degradation product, has been extensively used in clinical detection of coagulation disorders. A DD value less than 0.55 mg/L FEU is usually considered normal detected by means of immunoturbidimetry. DD has received growing attention since the outbreak of the coronavirus disease 2019 (COVID-19) pandemic, because of its pathological deterioration with the aggravation of cytokine storms, thrombosis, and disseminated intravascular coagulation (DIC) [5].

Aging is associated with the elevation of plasma levels of a wide variety of molecular markers, including DD, during coagulation activation [6]. In addition, increased DD levels are commonly found in various clinical settings such as inflammation, congestive cardiac failure, pneumonia, septicemia, terminal cancer, surgical procedure, pregnancy, and advanced age [7]. Further studies have taken DD as a potential indicator for its correlation with the prognosis of COVID-19, as well as community-acquired pneumonia in multiple studies [8]. However, little research has delved into the correlation of DD with patient prognosis, especially in the old population. Therefore, the motivation and novelty of the study is to explore the connection between DD and prognosis in shock and perioperative populations over 65 years of age.

## 2. Materials and Methods

### 2.1. Study Design and Research Population

This single-center retrospective study included 9,261 old patients ( ≥65 years of age) with either confirmed shock or in perioperative period of high-risk surgery hospitalized between January 2013 and December 2021 in ICUs of the Peking Union Medical College Hospital, a top tertiary hospital in China. We defined the study population because perioperative patients and septic shock patients were the most common populations with coagulation abnormalities in the ICU. Participants were either discharged or died prior to data acquisition.

### 2.2. Data Collection

We obtained demographic, clinical, laboratory, medication, and outcome data from the electronic medical records system for analysis. Demographic data covered gender, age, activity of daily living scale, etc. Laboratory results included blood routine examination, coagulation function related parameters (e.g., DD, fibrinogen, thromboplastin time, activated partial thromboplastin time, prothrombin time, prothrombin activity, and fibrin degradation products), inflammatory cytokines (ICs) on ICU admission (e.g., interleukin [IL]-6, C reactive protein [CRP], serum ferritin, procalcitonin, erythrocyte sedimentation rate [ESR], and lactate dehydrogenase), other assessments (hepatorenal function, myocardial enzymes and electrolytes), and multiple blood gas analyses. In our hospital, DD was measured using immunoturbidimetry. A DD level within the range of 0-0.55 mg/L FEU was considered normal. Clinical and medication data included outcomes, antibiotics, vasopressors, operations, ventilation time (VT), and length of ICU stay. The testing frequency was adjusted based on disease progression as assessed by the attending physician. Personal information was removed to protect privacy. Two physicians independently extracted the data using a standardized collection. Data accuracy was reviewed and confirmed by a third physician. Approval from the ethics committee of Peking Union Medical College Hospital (S-K360) has been obtained for this research, and all procedures were in compliance with relevant guidelines and regulations.

### 2.3. Endpoints

The primary endpoint was in-hospital mortality, while the secondary ones included length of ICU stay and VT.

### 2.4. Statistics and Analysis

The continuous data were denoted by median (interquartile range [IQR]) because none of them are normally distributed after the Kruskal-Wallis test. Categorical variables, tested by the Chi-square or the Fisher's exact test, were presented as number of cases (percentages). Mortality conforms to the Poisson distribution because it is a relatively low probability event. Multivariant analysis was performed using the Generalized Linear Model. Model 1 was univariant analysis. Model 2 was adjusted for gender, age, and the Sequential Organ Failure Assessment (SOFA) score according to previous study [9] and our preliminary analysis. Model 3 was adjusted for gender, age, SOFA score, operation, shock (defined as lactate increased with requirement for vasopressors), and antibiotics. The significance level was *p* < 0.05. All data was processed by SPSS 26.0 (IBM Corporation, Armonk, NY, USA).

## 3. Results

### 3.1. Demographic and Clinical Features

In general, 9261 patients were finally included, with 5026 (54.3%) of them being males; as to the age groups, 5145 (55.6%) and 3368 (36.4%) aged 65-74 and 75-84, respectively, while only 748 (8%) were very old patients (VOPs, ≥85 years old). DD elevations were common, with 89.9% of the tested patients above the upper limit of normal (ULN). 6288 (67.9%) of them had undergone operation, almost half were treated with antibiotics, and around one third were diagnosed with shock. The median SOFA score was 4 in the studied population.

In terms of the outcomes, 129 died in hospital. Most patients stayed in ICU for no less than 2 days. The median VT was 14 hours. See Table 1 for details.

### 3.2. DD Level on ICU Admission and Correlation with Serum Biomarkers

8813 of the patients had the DD level tested on ICU admission, with a median DD value of 2.18 mg/L (reference range 0-0.55 mg/L) and a normal DD found in only 975 (11%). Among those with an abnormal DD, 17.6% of them were between 1 and 2 ULN, 21.9% were between 2.1-4 ULN, 20.9% were between 4.1-8 ULN and 28.6% were more than 8 ULN (Table 2). Pearson correlation analyses were conducted among potential correlated factors, such as platelet (PLT), lactate dehydrogenase (LDH), DD, lymphocyte (L#), and white blood cells (WBC), by referring to previous research [9]. The correlation coefficient is listed in Table 2. As indicated by Table 3, statistical significance is present between DD and PLT, Fibrinogen, L# and WBC, but the correlation is relatively low.

### 3.3. DD Level at ICU Admission and Correlation with in-Hospital Mortality

Univariant analysis (Model 1) showed that higher DD levels were linked to a higher possibility of death (risk ratio [RR], 1.014; 95% confidence interval [CI], 1.009-1.020). However, after adjusting for demographics and SOFA score (Model 2), the associations became insignificant (RR, 1.005; 95% CI, 0.998–1.012). Nonsignificant significance was found in Model 3 (RR, 1.006; 95% CI, 0.998–1.014). (Figure 1).

Sensitivity analyses were performed for various age groups, gender, antibiotics, operation, and shock. All models were adopted. No statistical significance was found between the above factors and in-hospital mortality in these analyses. (Figure 2).

### 3.4. DD Llevel at ICU Aadmission and Ccorrelation with Llength of ICU Sstay

Model 1 showed that higher DD levels were correlated with longer ICU stay (RR, 1.066; 95% CI, 1.049-1.083). Model 2 slightly attenuated these associations (RR, 1.047; 95% CI, 1.030-1.065). The associations become insignificant in Model 3, a further adjusted model (RR, 1.012; 95% CI, 0.997–1.028). (Figure 1).

Sensitivity analyses showed interesting results. Taking Model 3 as an example, people who were between 65 and 74 years old (RR, 1.023; 95% CI, 1.003–1.043), without antibiotics (RR, 1.007; 95% CI, 1.001–1.013) nor shock (RR, 1.011; 95% CI, 1.002–1.021), but with surgical procedures (RR, 1.030; 95% CI, 1.012–1.048) were correlated with a longer ICU stay. While a correlation between a higher DD level and a shorter ICU stay was determined in VOPs (RR, 0.936; 95% CI, 0.888–0.985). There was no statistical significance in those aged between 75 and 84 (RR, 1.027; 95% CI, 0.996–1.058). (Figure 3).

### 3.5. DD Level on ICU Admission and Correlation with VT

Univariant analysis showed that higher DD levels were associated with longer VT (RR, 3.364; 95% CI, 2.563-4.417). Model 2 slightly attenuated these associations (RR, 2.666; 95% CI, 2.007-3.541), and Model 3 further attenuated these associations (RR, 1.577; 95% CI, 1.024-2.064). (Figure 1).

In Model 3, higher DD levels in females (RR, 1.804; 95% CI, 1.116-2.602), those who used antibiotics (RR, 1.736; 95% CI, 1.092-2.453), and those with operation (RR, 1.640; 95% CI, 1.273-2.114), and those with shock (RR, 1.740; 95% CI, 1.001-2.687) had a stronger correlation with longer VT than their counterparts. Those aged between 65 and 74 also showed a strong correlation (RR, 2.166; 95% CI, 1.491-2.864), while neither VOPs nor those between 75 and 84 had correlations with VT. (Figure 4).

## 4. Discussion

This is the first ever study investigating the impact of DD elevations on outcomes of the old population hospitalized in ICUs. Although DD levels were found to have no positive correlations with in-hospital mortality and length of ICU stay, they were strongly correlated with VT. Higher levels of DD in females, those who used antibiotics, those with operation and shock had stronger correlation with longer VT than the counterparts. Interestingly, the VOPs showed different trends from the younger age groups. Patients who were between 65 and 74 years old, without antibiotics, had undergone surgical procedures or without shock were correlated with a longer ICU stay.

### 4.1. DD Level and Clinical Outcomes

DD elevation, which represents the activation of coagulation and fibrinolysis systems, has been indicated as one of the most commonly seen laboratory abnormalities, as can be seen in malignant diseases, postoperative conditions, inflammation and infections [10]. DD had not been widely recognized as a prognostic biomarker until the COVID-19 pandemic. However, recent studies have reported higher DD levels in severe COVID-19 patients compared with mild counterparts [11]. A meta-analysis of COVID-19 patients showed that upregulated DD on admission is correlated with an evidently elevated possibility of all-cause death (RR, 4.77; 95% CI, 3.02–7.54) [12]. A DD level of 0.5 *μ*g/ml on admission was recommended as the cutoff for the risk of death for COVID-19 patients.

In our study, statistical significance was found between DD and VT, but not between DD and mortality or length of ICU stay. There might be some possible mechanisms for the close relationship between VT and DD. The entire lung vascular system is covered by the endothelial surface layer, which is responsible for vascular homeostasis [13]. For both perioperative and septic shock patients, inflammation can lead to increased levels of endothelial dysfunction that induces a prothrombotic state, resulting in relatively high incidence of lung injury in both groups [14, 15]. At the same time, endothelial dysfunction has been demonstrated to lead to prolonged ventilation [16], which in turn causes the reduction of endothelial cell density, thus prolonging VT and inducing more severe endothelial cell loss [17]. DD bind to endothelial cells though a series of receptors, such as ICAM-1 and integrins. It has been demonstrated that DD levels increased during inflammation, which suggested the presence of micro and macrovascular thrombosis in arteriovenous circulation [18]. Thrombotic complications were observed in 31% of ICU patients with COVID-19 infections [19]. There is also research reporting elevated DD and fibrin degradation products, as well as increased prothrombin time and activated partial thromboplastin time in COVID-19 nonsurvivors [20]. The rise in DD has been shown to be positively related to fibrin accumulating in the alveoli as a result of lung injury [21]. So, it is reasonable that higher DD levels led to longer VT, which is also a good explanation for the correlation between increased DD levels and longer length of ICU stay.

After adjusting for age, gender and SOFA, DD alone had little impact on mortality. Sensitivity analyses showed statistical significance in none of the groups, which was different from the recent studies conducted on COVID-19 patients [20, 22, 23]. According to an observational cohort study, biomarkers of epithelial cell damage and acute-phase proteins (soluble receptor for advanced glycation end-products [sRAGE], soluble tumor necrosis factor receptor 1 [sTNFR-1], etc.), rather than endothelial dysfunction-associated biomarkers, were linked to COVID-19 critical illness [24]. Further studies are warranted to explore whether epithelium or endothelium plays a dominant role in disease severity. And epithelial-associated biomarkers on mortality should be explored if the association between epithelial cells and disease severity is confirmed.

### 4.2. DD Level and the Impact of Aging

This study focused on the old population, because the median age of the entire ICU population may be already above 65 years as the population ages. The VOP population may be the fastest growing subgroup among ICU patients. And until recently, most ICU physicians have been reluctant to admit these VOPs. The outcomes for this group may be different from the younger counterparts [25]. Unlike many previous studies, our study fails to demonstrate a correlation between DD and the outcomes of VOPs [26, 27]. We even concluded that DD elevations were linked to a shorter ICU stay in VOPs in Model 3, which is hard to explain and may be attributed to a number of factors. Only 19 out of the 749 VOPs died in hospital, which can demonstrate that the admission and discharge policy for VOPs are more flexible in clinical activities. The average SOFA score of the VOPs was 4.08 (standard deviation [SD], 3.55), which means that these VOPs are highly feasible for the study; they consented to risky procedures; anesthetists and surgeons agree to perform the surgeries, and very few VOPs have limitations on life-support treatment [28, 29]. Most of the VOPs did not undergo major surgery or experienced severe septic shock. Several factors like end-of-life decisions and ICU quality of care also influence their outcomes. All the above “confounding factors” affect the ultimate result. Another possible explanation is that higher DD levels mean more severe endothelial dysfunction [30], which means more severe disease and shorter time to outcome. While in patients aged 65-74, both the reaction and the therapy were more similar to those aged 18-64. The results might be more reasonable.

### 4.3. DD Level and the Impact of Antibiotics, Surgery Procedure and Shock

In previous studies, multiple factors, such as old age, male, shortness of breath, hypertension, diabetes mellitus, coronary heart disease, cerebrovascular disease, gastrointestinal reactions, psychiatric symptoms, renal dysfunction, and traumatic fractures have been confirmed to affect DD levels and patient outcomes [31]. In this study, we proved that higher DD levels in females, those who used antibiotics, those with operation, and those with shock had a close correlation with longer VT than the counterparts. The results are reasonable, as infections, operation, and shock are all risk factors that promote inflammation that aggravates endothelial injury. (1) All kinds of infections can cause the release of pro-ICs, including IL-2, IL-6, IL-7, MCP-1, and TNF-*α* [32]. This is followed by high activation of macrophages, T cells, and natural killer cells, releasing more than 150 kinds of ICs [33]. Endothelial cells become dysfunctional when there is a cytokine storm, leading to an abnormally activated coagulation system [34]. (2) Surgery itself is a stress response as well as a general inflammatory response that promotes the production of catecholamine and glucocorticoid [35]. Stress response also includes sympathetic activation and increased shear stress on the vessel wall. A systematic review on endothelial dysfunction after noncardiac surgery showed immediately decreased endothelial function after surgery, which might be improved 1 month later [36]. (3) In shock patients, hypoperfusion, microcirculation impairment, and endothelial dysfunction promote each other, with endothelial dysfunction playing a vital part in hemodynamic homeostasis imbalance. All the above factors can affect the DD levels, as well as VT [37]. In conclusion, infection, operation, and shock are the risk factors for prolonged VT.

In this paper, we also determined that in noninfection, nonshock, and operation patients, DD elevations were correlated with length of ICU stay. Although insignificant, the infection group has a higher RR than the noninfection counterpart. This is similar to the interpretation for VT above.

### 4.4. Limitations of the Study

The study has several limitations, though it has a relatively large sample size. While some correlations have been found through statistical analyses in this single-center retrospective study, the results obtained require larger-scale validation. We believe that the correlation between DD levels and patient outcomes is related to the endothelial dysfunction caused by multiple factors, but we have not tested that theory. In the future, we will design prospective studies to verify this hypothesis. Second, only DD levels at the time of ICU admission were available. As a result, we were unable to assess alterations in DD levels over time, let alone the impacts of these alterations on clinical outcomes. Third, as we mentioned above, the admission and discharge policy are more flexible in clinical activities with age, which improved individual heterogeneity. Clinical studies aimed that VOPs may address this issue.

## 5. Conclusions

Elevated DD levels at ICU admission are linked to an increased risk of VT and prolonged length of ICU stay in the old population with either confirmed shock or after high-risk surgery, indicating the potential role of DD as a warning sign to predict disease severity, as well as a marker of prognostic utility for all ICU patients in the future.

## Figures and Tables

**Figure 1:** DD levels at ICU admission and correlation with mortality, length of ICU stay and VT. DD: D-dimer; VT: ventilation time.

**Figure 2:** Sensitivity analysis of DD levels at ICU admission and correlation with mortality. DD: D-dimer.

**Figure 3:** Sensitivity analysis of DD levels at ICU admission and correlation with length of ICU stay. DD: D-dimer.

**Figure 4:** Sensitivity analysis: DD levels at ICU admission and correlation with VT. DD: D-dimer; VT: ventilation time.

**Table 1:** Demographic and clinical characteristics (including D-dimer level) of the study population.

ITEM	*N*	%
AGE		
65-74	5145	55.6
75-84	3368	36.4
≥85	748	8
Gender		
Male	5026	54.3
Female	4235	45.7
Operation		
Yes	6288	67.9
No	2973	32.1
Shock		
Yes	3069	33.1
No	6192	66.9
Antibiotics		
Yes	4913	53.1
No	4348	46.9
D-dimer		
Normal	975	11.1
1-2 ULN	1546	17.6
2.1-4 ULN	1928	21.9
4.1-8 ULN	1837	20.9
>8 ULN	2523	28.6
Mortality	129	1.4

Note: ULN: upper limits of normal.

**Table 2:** Demographic, serum biomarkers and clinical features of the study population.

	N	Minimun	25th percentile	Median	75th percentile	Maximun
Age	9261	65	69	73	79	105
D-dimer	8813	0.2	0.99	2.18	4.83	297.2
L#	9183	0	0.49	0.73	1.12	29
SOFA score	8763	0	1	4	7	21
Length of ICU stay	9261	1	2	2	4	248
Ventilation time	7004	1	7	14	21	2637

Note: L#: lymphocyte count; SOFA: Sequential Organ Failure Assessment.

**Table 3:** Pearson correlation analyses among serum biomarkers.

	PLT	LDH	Fibrinogen	D-dimer	L#	WBC
PLT	1	-0.041	0.357^∗^	-0.078^∗^	0.16^∗^	0.138^∗^
LDH		1	-0.068	0.036	0.057	0.009
Fibrinogen			1	0.051^∗^	0.032^∗^	0.09^∗^
D-dimer				1	-0.004	0.07^∗^
L#					1	0.142^∗^
WBC						1

Note: Bold text indicates the presence of statistical significance. PLT: platelet; LDH: lactate dehydrogenase; L#: lymphocyte; WBC: white blood cells. ^∗^ *P* < 0.05.

## Data Availability

Data and materials are available from the corresponding author on reasonable request.
